This article has been retracted.

# Sensory Coding by Cerebellar Mossy Fibres through Inhibition-Driven Phase Resetting and Synchronisation

**DOI:** 10.1371/journal.pone.0026503

**Published:** 2011-10-26

**Authors:** Tahl Holtzman, Henrik Jörntell

**Affiliations:** 1 Behavioural and Clinical Neuroscience Institute and Department of Experimental Psychology, University of Cambridge, Cambridge, United Kingdom; 2 Section for Neurophysiology and Neuronano Research Center, Lund, Sweden; Tokyo Medical and Dental University, Japan

## Abstract

Temporal coding of spike-times using oscillatory mechanisms allied to spike-time dependent plasticity could represent a powerful mechanism for neuronal communication. However, it is unclear how temporal coding is constructed at the single neuronal level. Here we investigate a novel class of highly regular, metronome-like neurones in the rat brainstem which form a major source of cerebellar afferents. Stimulation of sensory inputs evoked brief periods of inhibition that interrupted the regular firing of these cells leading to phase-shifted spike-time advancements and delays. Alongside phase-shifting, metronome cells also behaved as band-pass filters during rhythmic sensory stimulation, with maximal spike-stimulus synchronisation at frequencies close to the idiosyncratic firing frequency of each neurone. Phase-shifting and band-pass filtering serve to temporally align ensembles of metronome cells, leading to sustained volleys of near-coincident spike-times, thereby transmitting synchronised sensory information to downstream targets in the cerebellar cortex.

## Introduction

Oscillatory neuronal activity is considered fundamental for enabling co-ordinated activity during normal brain functioning [1]–[3] whilst disturbances of oscillatory activity are associated with a variety of brain disorders including epilepsy, Parkinson's disease and schizophrenia [4], [5]. In general, oscillogenesis is considered to arise from the concerted interplay of excitation and inhibition within a local network [for review see 6], [7], although intrinsic oscillatory behaviour can also operate at the single neurone level. Electrical coupling and intrinsic membrane currents may interact to produce prominent oscillatory activity, such as that seen in cells of the inferior olive [8], [9], prompting the suggestion that synchronous oscillations provide a temporal reference for control of motor performance. Passive and active membrane conductances can bias cells to oscillatory activity at preferred, resonant frequencies [reviewed by 10]. For example, cerebellar granule cells and Golgi cells show a low frequency resonance [11]–[13] suggesting that they may be tuned to respond to oscillatory afferent signals in a narrow frequency range.

At the cellular level, representation of information using oscillatory schemes gives rise to phase-of-firing coding, where neurones fire at particular times during an on-going oscillation thereby implementing a temporal code [see 14]. Sub-threshold oscillations, and thus spike-time reliability, can be phase shifted by excitatory inputs [15], [16] and by inhibitory inputs [17]–[19] suggesting that oscillatory information coding can adapt dynamically. Downstream neurones must be able to read-out such codes and might employ a variety of mechanisms including spike counts and spike-time dependent plasticity [see 20]–[23]. In this regard, cortical neurones are well-suited to detect correlated oscillatory activity [24] as are the much smaller, electrotonically compact cerebellar granule cells [25], [26].

In this study we examine a novel class of neurones located in the lateral reticular nucleus of the brainstem, whose axons form a major supply of afferents to the cerebellar cortex [27]. These units fire with remarkable regularity at idiosyncratic frequencies ranging from ∼7–22 Hz. Sensory evoked inhibition serves to phase reset their regular spike firing enabling spike-time locking to particular sensory stimulation frequencies. Using phase-response curves, joint-peristimulus time histograms and simulations we show that phase resetting can generate synchronised volleys of near-coincident firing capable of representing a temporal code of sensory input frequency that is well-suited to influence downstream neurones such as Golgi cells and granule cells in the cerebellar cortex.

## Materials and Methods

Experiments were performed, in vivo, on 50 adult Wistar rats weighing 300–450 g. All procedures were conducted so as to minimise suffering and were approved by the local ethical review panel of the University of Cambridge and by UK Home Office regulations (Project number 80/2234). The methods for general preparation have been described previously [28]. Under urethane general anaesthesia (1–1.5 g/kg i.p.) supplemented with 0.1 ml Hypnorm (i.p.) rats were fixed in a stereotaxic frame and the cerebellum was exposed. Single unit recordings were made from units located in lobules Crus Ic/II a/b and in some experiments recordings were also obtained from the lateral reticular nucleus (LRN) in which the foramen magnum was opened, exposing the brainstem landmark obex. For cerebellar penetrations electrode angles were ∼45 degrees from vertical so as to be perpendicular to the cerebellar folial surface; depth from surface rarely exceeded 700 µm and crossing of Purkinje cell layers was carefully determined in each electrode track. LRN recordings were targeted using stereotaxic co-ordinates [29] – electrode angle 30 degrees from vertical, interaural −4.2 mm AP, interaural −0.3 to −0.5 DV and midline +1.9 mm, following the histologically verified approach of [30]. Signals from the microelectrodes were amplified (gain ×1000–10000), filtered (band-pass 0.3–10 kHz for spikes and 0.1–300 Hz for local field potentials [LFP]) and digitised at 25 kHz (spikes) and 5 kHz (LFP). Some recordings were made using platinum/tungsten electrodes coated with quartz glass – 80 µm shaft diameter – impedance 2–3 MΩ Thomas Recording - Giessen, Germany) arranged in a 4×4 array or concentric 6+1 array (Eckhorn & Thomas, 1993) whilst on other occasions we used glass micropipettes pulled from filament glass broken to give tip impedances of 6–15 MΩ when filled with 0.5 M NaCl.

During LRN recording experiments, a stainless steel stimulation electrode (100 kΩ, Microprobes, MD 20879, USA) was inserted into the cerebellar cortex/white matter. Biphasic stimulus pulses (0.2 ms, 2 Hz, 100–400 µA) were used to elicit antidromically activated spikes in LRN units with all-or-none characteristics and constant latency (typically ∼1.5 ms). Since all of our units were spontaneously active, antidromicity was confirmed by cancellation of evoked spikes by collision with spontaneously occurring spikes (Figure 1B), confirming the identity of these LRN units as cerebellar-projecting mossy fibres.

**Figure 1:** Spontaneous firing properties of metronome cells. **A** shows a 5 second excerpt of spontaneous spiking activity from an example metronome cell recorded in the brainstem, alongside the superimposed spike waveforms. **B** plots the ISIH for this neurone which had an idiosyncratic frequency ∼13 Hz (bin size 1 ms). The *inset* shows 10 traces of raw data where spontaneous spikes were used to trigger delayed antidromic stimulation in the cerebellum. In the *upper* traces, antidromically evoked spikes occur at fixed latency (1.3 ms). When stimuli are triggered at less than this latency, no antidromic spikes are evoked (*lower* traces indicated by * - stimulus delay 1 ms) due to collision with spontaneous orthodromically conducted spikes. Similar data for an example cerebellar metronome unit (slower idiosyncratic frequency ∼8 Hz) are plotted in **C** and **D**. Group data for mean firing frequency and CV2 calculated from spontaneous activity of brainstem and cerebellar units is plotted in **E** (note that whilst all units were spontaneously active, records of spontaneous activity were obtained from a subset of our sample). No significant differences were found between these groups comparing either parameter. **F** plots CV2 for a variety of neurones in the cerebellum and the neocortex, indicating that metronome cells are particularly regular.

Mixed low-threshold somatosensory afferents were stimulated using percutaneous pin electrodes inserted in to the foot pads and vibrissal skin at rates generally <0.66 Hz. During some experiments we used trains of stimuli at frequencies ranging from 6–30 Hz, with trains lasting for ∼1000 ms or 500 ms (frequencies >20 Hz). Spike trains were discriminated using a custom written spike shape analysis and cluster-cutting package (LabSpike, Dr. Gary Bhumbra, Dept. of Physiology, Development and Neuroscience, Downing Street, Cambridge, UK; available from http://www.pdn.cam.ac.uk/staff/dyball/labspike.html) and the time series were used to construct peri-stimulus time-histograms (PSTHs) and interspike interval histograms (ISIHs). Phase response curves for somatosensory input were calculated for some metronome cells, using stimuli delivered at random relative to the spontaneous firing. Prior to each stimulus, a period of spontaneous firing (typically 5–6 spikes) was used to estimate the time of the expected spike if no stimulus had occurred, thus perturbation phase was calculated using the time of the expected spike and its predecessor, taking into account peripheral conduction delays (∼10 ms; estimated from the PSTH).

To assess spike-time accuracy during stimulus trains we calculated a spike-stimulus synchronisation index (SI), by treating the time interval between stimulus pulses with a periodic function, thus:where *h_i_* = number of spikes occurring in the *i^th^* phase bin of *n* (typically 36 bins, corresponding to 10 degrees per bin).

ISI distributions were expressed as probability density distributions using a kernel density estimation algorithm [31] allowing grouping of datasets and normalisation for idiosyncratic frequencies of individual cells. Spike triggered averages of LFP (STA-LFP) were constructed by taking epochs of LFP, typically 100 ms either side of each spike. Confidence limits were calculated using Monte Carlo simulations (spike-times and LFP segments shuffled, minimum 100 simulations). Coherence between spikes and LFP was calculated using spike-field coherence (SFC) as detailed by [32] and Monte Carlo simulations were used to generate confidence bounds (1000 simulations). For metronome cell ensemble recordings we used the joint-peristimulus time-histogram (JSPTH) technique to assess time-resolved stimulus-evoked correlations between cell pairs [33]. JPSTHs were constructed using 2 ms time-bins and smoothed using a gaussian where σ = 2 ms.

A simple model of granule cell synaptic integration, similar to that used in our earlier work [25], [26], was used to calculate the summation of mossy fiber-EPSPs. The only purpose of this model was to analyze the pattern of membrane potential fluctuations, which could be obtained as a result of varying the number and temporal density of synaptic inputs. In granule cells *in vivo*, the spike output is essentially a linear function of the membrane potential [25], so these membrane potential fluctuations should be closely correlated to spike output, although this remains to be confirmed in actual recordings from granule cells receiving inputs from this type of LRN cell. In this paper, we set the model to operate at a membrane potential of −59 mV to prevent spiking. The model assumes that different mossy fiber synapses have different average EPSP amplitudes [25]. As the model was used for simulations within a narrow membrane potential range, it was simplified to not include any active membrane conductances or Golgi cell inhibition. Time-courses and amplitudes of each mossy fiber-EPSP (at −59 mV) and the paired-pulse depression ratio when an individual mossy fiber input is activated at high rates were based on data for the mossy fiber-EPSPs *in vivo* [25]. The following parameters were used for the EPSPs: EPSP peak amplitudes at 800 MΩ (membrane resistance for granule cells in vivo) (synapse 1–4): 5.2; 4.0; 3.2; 2.5 mV; time-to-peak: 0.95 ms; half-time decay: 5.5 ms; paired-pulse depression, max. 63% (at 1 ms interval); paired-pulse depression time constant: 8 ms. The spike responses, recorded at a temporal resolution of 0.1 ms, of single metronome cells were fed to each of the four mossy fiber inputs.

## Results

### Metronome-like activity in LRN cells

We made recordings from brainstem units (n = 41, 15 animals) located in the lateral reticular nucleus (LRN) and also from mossy fibre terminals in the cerebellar cortex (n = 70, 35 animals). All of these units were spontaneously active (i.e. in absence of overt sensory stimulation) and their firing patterns were distinctive in their regularity. The raw spike train and interspike interval histogram (ISIH) shown in Figure 1A and 1B show data from an example LRN unit with a mean firing rate of ∼14 Hz. We only included units recorded in the LRN which were positively identified as cerebellar-projecting using antidromic collision testing (see Methods). Example collision data are shown inset in Figure 1B. Across the population of cells tested, collision latencies ranged from 1.1–1.9 ms, consistent with fast-conducting fibres (c.f. ∼5 ms climbing fibre conduction latency from the inferior olive [34]). In other experiments, we recorded units with similar firing patterns in Crus I/II of the cerebellar cortex. An example unit is illustrated in Figure 1C and 1D. The action potential waveform of this unit (and all others like it recorded in the cerebellum – see also Figure S1C and S1D) comprised an early fast- and later variable slow-component typical of mossy fibre terminals [25], [35]–[37]; the fast component represents the axonal action potential and the slow, variable amplitude component (negative after-wave; NAW) reflecting elements of the synaptic action potential and post-synaptic response. Such units were commonly encountered alongside spikes belonging to Golgi cells and granule cells [see 28], [38].

Comparing LRN units with cerebellar units, their mean firing rates and the regularity of their firing patterns [measured using CV2; 39] are plotted in Figure 1E, for a selection of units from each population. Across our sample, individual units fired at a range of idiosyncratic mean frequencies ranging from ∼7–22 Hz; the distinct regularity of these firing patterns generated CV2 values which were generally <0.13 - moreover, our brainstem neurones showed highly similar characteristics when compared to those units recorded in the cerebellum (Figure 1E). A one way multivariate analysis of variance test did not find evidence of a significant difference between these two groups (p<0.1494) consistent with these samples being drawn from the same underlying population. Metronome cells appear to be the most regular firing of cell types in the cerebellum (perfect regularity generates CV2 = 0) compared to other cell types such as Purkinje cells, Golgi cells and granule cells [28], [40], [41], and in comparison to neocortical cells [39] (Figure 1F).

In summary, the similarity of the cerebellar metronome firing patterns to those in the brainstem alongside their dissimilarity to other cerebellar cortical neurones in the granular layer considered along with action potential waveforms characteristic of mossy fibres (see also insets in Figure S1 – see also identical response patterns between cerebellar and brainstem unit), make it likely that our sample of cerebellar units represents the synaptic terminals of metronomic LRN neurones, none-the-less in the absence of definitive proof, our classification remains putative.

The highly regular firing patterns of metronome cells could arise via intrinsic oscillatory currents, network activity or regular afferent inputs – these scenarios are not mutually exclusive. We used spike-triggered averaging (STA) of local field potentials (LFP) recorded in the LRN to address this question. LFP-STAs are useful for assessing the relationship between spikes (supra-threshold) and peri-spike membrane activity (sub-threshold) since the LFP represents the average of both supra- and sub-threshold events from a volume of several 100 µm [for review see 42]–[45].

Example STAs calculated for a pair of simultaneously recorded LRN units (different electrodes) are drawn in Figure 2A and 2B. Peri-spike periodic voltage oscillations dominate the STA; the period of these oscillations closely matches idiosyncratic firing frequency of each cell, 16 Hz and 12 Hz, respectively. All LRN STA's showed peri-spike periodic voltage oscillations (n = 6). We used a *Monte Carlo shift predictor* (spike times randomised, STA recomputed; 100 shuffles - superimposed broken grey lines) to calculate 95% confidence interval for the STA, thus values exceeding these bounds (grey lines) are considered significant (p<0.05). This neurone pair was separated by approximately 300 µm – we also computed the STA using spikes from one cell and the LFP signal from its counterpart, giving rise to a ‘flat’ STA (Figure 2C). Similar results were obtained for other cross-referenced STAs using simultaneous recordings (data not shown). STA oscillations were typically 40–80 µV peak to peak, comparable in size to STA oscillations reported elsewhere in the brain [46]–[49]. These results suggest that peri-spike oscillations are generated focally (i.e. spatially restricted), rather than representing distributed network activity such as that seen during hippocampal theta oscillations [50].

**Figure 2:** Spike-LFP coherence of metronome cell firing. **A** and **B** show spike-triggered averages of LFP for two example metronome cells (recorded simultaneously on separate electrodes). In each case, spikes referenced to their own LFP signal revealed peri-spike periodic voltage fluctuations (solid lines). Monte Carlo based confidence limits (95%) are superimposed on each plot (broken grey lines). **C** shows the STA using spikes from the cell in **A** referenced to LFP of the cell in **B** using the same format – although recorded simultaneously and separated by ∼300 µm no relationship between spikes and LFP was apparent. **D** and **E** plot spike-field coherence (solid lines) for the same cell pair. Monte Carlo based confidence limits (95%) are superimposed on each plot (broken lines) along with probability density estimates for the spiking frequency of each cell (grey curves). Grouped data for SFC values (mean ±2 S.E.M.), normalised for idiosyncratic firing frequency are plotted in **F**.

We also calculated spike-field coherence (SFC) to assess phase synchronization between the LFP and spike times as a function of frequency [32]. SFC is a unitless measure between zero and one – values of one suggest a constant phase synchronisation of spikes with the LFP. Figure 2D and 2E show SFC spectra for each STA (solid lines) with maximal peak values at 0.66 and 0.37, respectively. Confidence limits were generated using Monte Carlo simulations (95^th^ centile of 1000 *shift predictors* – broken lines), thus SFC values above these limits are considered to be significantly above levels expected by chance synchronisations between spikes and LFP frequency components (p<0.05). Dominant peaks in the SFC spectra were closely linked to idiosyncratic firing frequency, c.f. superimposed spike frequency distributions (grey curves) in each example. Grouped data are plotted in Figure 2F (normalised for the idiosyncratic firing rate of each cell) which shows a 95% confidence interval for SFC values with respect to normalised idiosyncratic firing frequency; maximal phase synchronisation occurs at frequencies closely corresponding to the cell's idiosyncratic firing frequency. We conclude that peri-spike voltage oscillations and spike output are closely synchronised.

The localised origin, spike-time dependence and the spike field coherence for peri-spike periodic STAs suggests they represent membrane voltage fluctuations from the individual neurones under study. These findings are consistent with the regular firing patterns of metronome cells being underpinned by intrinsic oscillatory currents [44].

### Sensory evoked silent periods phase reset metronome cells

Somatosensory activation interrupted the regular firing of metronome cells by causing a brief silent period (duration 40–50 ms) following which the spontaneous spiking resumed, thus sensory evoked silent periods served to reset the spike-times of the regular spiking metronome cells (Figure 3A). Responses of this type could be evoked from widespread areas of the skin, including the face and limbs, and consistent with previous studies of LRN neurones [51], [52], metronome cells had widely convergent, often bilateral receptive fields (see Text S1 and Figure S1). In the example PSTH shown in Figure 3A, stimuli were delivered at random relative to the firing of the cell. Reorganising the raster based on the *expected* spike times (see Methods), reveals the phase response properties of this neurone (Figure 3B). Intuitively, many of the observed spikes following the perturbations are delayed (i.e. evoked silent periods extend the interspike interval = phase *pro*cession; trials 1∼30) whilst others show little or no deviation (trials 31∼50). However, the perturbation caused many spikes to occur *earlier* than expected (trials 51∼71: phase *pre*cession). A spike-time phase response curve (PRC) for this cell is shown in Figure 3C. The shape of the PRC is related to spike-generation mechanisms and thus offers a precise characterisation of the effect a perturbation has on an on-going oscillation and the timing of subsequent spikes [53]. The PRC shown in Figure 3C indicates that perturbations of the regular firing of this metronome cell occurring soon after spontaneously generated spikes (phase 0–0.3) tended to advance the subsequent spike-time by 5–10 ms (triangles <0). Spike-time delays up to 60 ms were observed for perturbations occurring later in the firing cycle. Given the idiosyncratic firing frequency of this cell was 12–13 Hz these changes in spike-time range from ∼10% advancement to ∼75% delay.

**Figure 3:** Somatosensory stimulation briefly silences and phase-resets metronome cell spike timing. **A** shows a PSTH (bin size 5 ms) and raster from an example metronome cell following sensory stimulation (limb stimulus, 0.6 Hz). Note the evoked silent period shortly after each stimulus (onset latency ∼10 ms, duration 40–50 ms) which stops the spontaneous spiking of the cell, thereby ‘resetting’ the subsequent spike-timings, evident as peaks in the PSTH. **B** shows the same raster as in **A** reordered by the expected spike-time (see Methods) for each trial (red triangles). The first observed spike-times after each stimulus are indicated by blue triangles – note the spike-time delays (*lower* half of panel) and spike-time advancements (*upper* half of panel). **C** plots the phase-response curve for this same cell, summarising the raster shown in **B**. The phase response curve in **D** show grouped data, normalised for idiosyncratic firing frequency; solid lines represent a 95% confidence interval for the median in each of 10 phase bins. The phase response curves in **E** and **F** extend the analysis to the subsequent interspike intervals (cf. green and pink triangles in **C**).

The PRC for group data from 18 cells tested in the same way (40 perturbations each) is shown in Figure 3D – data are normalised for idiosyncratic firing frequencies. Each triangle represents a perturbed spike-time from an individual cell (cf. blue triangles in Figure 3B). Data are grouped into 10 phase bins with 95% confidence intervals calculated for the mean of each bin (solid lines). The PRC indicates that for a typical metronome cell, phase advancement of 5–10% is likely to occur for perturbations that arrive within the first third of a typical firing cycle (i.e. observed spike-times are 5–10% earlier than expected). Little or no change in spike-time was apparent for perturbations delivered across 30–40% of a ‘typical’ firing cycle, whereas for all later-arriving perturbations subsequent spike-times were delayed by up to 50%.

We extended the analysis to the 2^nd^ and 3^rd^ spike-times in the series (green and pink triangles, respectively in Figure 3B). We found that the adjacent interspike interval (2^nd^ spike) tended to show a modest spike-time advancement of 5–10% (Figure 3E, cf. Figure 3B), irrespective of the phase of the initial perturbation. The spike-times of the 3^rd^ (and subsequent spikes – not shown) did not show this effect. This finding indicates that the influence of the evoked silent periods may extend to 1^st^ and 2^nd^ spike-times after the perturbation, but not beyond.

The spike-time advancement arising through presumed inhibitory input (i.e. evoked silent periods) suggests that inhibition-activated depolarising mechanisms, such as *Ih* [54], might be brought into play following sensory input. Metronome cells can thus reflect the precise timing of sensory events by the phase response of their spike-time resetting, on a trial-by-trial basis.

### Spike-time alignment of metronome cell firing to rhythmic sensory input patterns

The regular firing pattern of metronome cells at idiosyncratic frequencies ranging from ∼7–22 Hz prompted us to examine the effects of rhythmic somatosensory stimulation on spike-timing. We used trains of stimuli ranging from 6–30 Hz; a bandwidth that encompasses rhythmic movements such as licking, grooming, locomotion and also the distribution of idiosyncratic firing rates of metronome cells (Figure 1E).

Metronome cells showed a pronounced ability to stimulus-lock their spike times across a broad range of sensory stimulation frequencies. Data from an example cell are shown in Figure 4. Ascending stimulation frequencies (2 Hz steps) cause pronounced shifts in the overall activity of this cell (cf. Figure 3C), as shown by the close relationship between spike-times and individual stimulus pulses (black triangles – Figure 4A). During sensory stimulation, spike firing shifted toward the stimulation frequency; this cell was able to lock onto input frequencies <10 Hz (cf. ISI probability distributions, Figure 4B), whilst for input frequencies 10–16 Hz, the firing was split into at least two distributions each tending toward the stimulation frequency or half of this value, respectively. With increasing stimulation frequency, spike firing became increasingly locked to half of the stimulation frequency, reaching a ceiling at >24 Hz, where the stimulus-locking relationship broke down. In order to assess spike-time alignment precision at different input frequencies, we calculated a spike-stimulus synchronisation index (SI – see Methods; Figure 4C). This provided a unitless measure between 0 and 1, thus if all spikes occur at the same phase relative to each stimulus pulse, SI = 1. In this particular example, spike-stimulus synchronisation exceeded 0.5 for frequencies in the range 8–20 Hz, thus at least half of the spikes had a consistent relationship to the stimulation frequency; this particular cell had an idiosyncratic frequency of ∼14 Hz. Given that stimulation could last for ∼1000 ms (see Methods), these findings indicate that metronome cells can show sustained spike-time alignment to a broad range of sensory input frequencies.

**Figure 4:** Rhythmic somatosensory stimulation entrains metronome cell spiking in a band-pass like manner. The PSTHs in **A** show the responses of an example metronome cell during a variety of rhythmic stimulation patterns (stimulus frequency indicated beside each PSTH, stimulus pulse times represented by solid triangles under each PSTH; bin-size 10 ms). Simple visual inspection of the PSTHs is misleading as it obscures trial-by-trial variability, thus we computed probability density estimates for the interspike interval frequencies (**B**) before and during the stimulus trains (white and black distributions, respectively). To aid visual inspection, in each plot in **B** stimulation frequency is indicated by the open triangles whereas the grey triangles represent half of this value – note the tendency for spiking frequencies to centre around these values at different stimulation frequencies. Spike-time accuracy with respect to each stimulus pulse in the train was calculated using a spike-stimulus synchronisation index (see Methods).

In order to group data across cells, we normalised for the idiosyncratic frequencies of our cells. Data for 12 cells tested with the range of input frequencies are plotted in Figure 5A, where the ISI frequency distributions during stimulation are represented as colour-coded probability density. Grouping the data in this way suggests that stimulus-locking (either at the stimulation frequency or half of this value) will occur for inputs in the range of 0.5 to <2-times the cell's idiosyncratic frequency, indicated by the diagonal trends in the colour plot (cf. Figure 4B). Grouped data for the spike-stimulus synchronisation index are plotted alongside (Figure 5B). Analogous to tuning curves and best-frequencies for auditory hair cells, maximal spike-time accuracy for individual cells occurs with input frequencies close to the idiosyncratic frequency.

**Figure 5:** Population entrainment in response to rhythmic somatosensory stimulation. A plots grouped data for 12 metronome cells tested with the gamut of rhythmic stimulation frequencies – data were grouped as probability density estimates and normalised for idiosyncratic firing rates, thus stimulation frequencies are expressed relative to these values for each cell. The diagonal trends in the probability density distributions indicate the tendency for the metronome cells to alias stimulation frequencies in the range of 0.5 - <2 times their idiosyncratic frequencies. **B** plots the spike-stimulus synchronisation index derived from the same grouped data, indicating that maximal spike-time accuracy with respect to individual stimulation pulses occurred for stimulation frequencies close to the idiosyncratic firing frequency. Data are plotted as mean ±2 S.E.M.

It is not straight-forward to interpret the PRC analysis alongside these findings, although it is noteworthy that on average, cells tend to decelerate (i.e. phase *delay*) and similarly they may also show modest acceleration (i.e. 5–10% phase *advance*) for input frequencies <1.5-times the idiosyncratic frequency, cf. white dotted line in Figure 5A. These findings suggest that across the population of metronome cells subsets of cells are capable of stimulus-locking to a broad range of input frequencies, consistent with individual cells performing a ‘band-pass’ operation similar to that seen in cortical and trigeminal neurones [55], [56].

### Sensory evoked silent periods drive correlated firing in metronome cells

Phase resetting of spike-times, and stimulus-locking during rhythmic sensory activation will have important consequences for the downstream target neurones; the cerebellar granule cells. Anatomical convergence and synchronisation of multiple metronome cells could transform relatively slow spike-trains (∼7–20 Hz across the metronome cell population) into high frequency, near-coincident, volleys of excitatory post-synaptic potentials – an essential requirement for spiking in granule cells [25], [26].

To assess time-resolved stimulus-induced correlations between simultaneously recorded metronome cells, we used the joint peri-stimulus time histogram technique [JPSTH – 33]. Our analysis suggests that the evoked silent periods following sensory stimulation can synchronise metronome cells, for the duration of the sensory stimulation. We analysed data from 11 LRN neurones (12 possible pairs recorded simultaneously) tested with a range of stimulation frequencies (see Figure 4). Assessment of the normalised JPSTHs (i.e. normal JPSTH minus shift-predictor) showed no residual correlations (data not shown) indicating that any correlations between metronome cells were underpinned by stimulus-induced spike-time changes, rather than arising through mutual connections [33]. Since we found no evidence for correlations other than those driven exclusively by stimulation, henceforth we only consider the bin-by-bin cross-product of the two PSTHs (‘predictor’, alternatively the PST-product) – this represents the null hypothesis that spiking probabilities are related to the stimulus, although each neurone fires independently of its counterpart. We first examined near-coincident firing arising from *single* stimuli – example data for a metronome cell pair are drawn in Figure 6A (idiosyncratic frequencies ∼12 Hz and 14 Hz, respectively). The main diagonal of the JPSTH gives rise to the ‘PST coincidence histogram’ (Figure 6B) which displays the observed rate at which both neurones fire simultaneously (to within the accuracy of the bin-width of the histogram – 2 ms). Near-coincident activity is most likely at ∼50 ms latency (i.e. the first spike following the evoked silent periods in each neurone). Subsequent near-coincident firing occurs due to stochastic interaction of the cells' idiosyncratic frequencies, producing the interference pattern visible in the correlation delay matrix (paradiagonal to JPSTH diagonal) shown in Figure 6C, which highlights the lead-lag times for near-coincident spike-timings. The arbitrarily chosen lead-lag range of −25 to +25 ms corresponds to a minimum instantaneous frequency of 40 Hz – if these metronome cells projected to the same granule cell, the principal coincidences for this cell pair would generate EPSPs at rates >200 Hz (taken as the instantaneous frequency of the spikes generated by the cell pair). Grouped data for 11 metronome cell pairs tested with *single* stimuli are shown in the same format in Figure 6D – thus, the population response of metronome cells (of differing idiosyncratic frequencies) following a single stimulus is a well synchronised, but brief lived increase in near-coincident firing at ∼50 ms (see expanded time-base in *lower* panel).

**Figure 6:** Near-coincident firing in metronome cells induced by single somatosensory stimuli. **A** shows the JPSTH for a pair of simultaneously recorded metronome cells following a single sensory stimulus (limb); the matrix represents the PST-product, from which the diagonal is used to give rise to the PST coincidence histogram shown in **B**. A further extension of this is the correlation delays matrix shown in **C**, which highlights epochs of near-coincident firing for the cell pair, along with lead-lag times between counterpart spikes corresponding to a minimum of 40 Hz. Note that near-coincident firing is most probable ∼50 ms after the stimulus onset (i.e. latency of the first phase-reset spike-time) with subsequent stochastic interactions between the cells as they resume their idiosyncratic firing patterns (see Figure 3). The correlation delay matrix shown in **D** plots grouped data for 11 cell pairs tested with single sensory stimuli. **E** plots correlation delay matrices for the same cell pair illustrated in **A**–**C**, during a variety of rhythmic stimulation patterns – stimulation frequency is indicated besides each panel, and individual pulse times are represented by vertical white lines. Lead-lag times in each panel are 0±25 ms (arbitrarily chosen), corresponding to a minimum instantaneous frequency of 40 Hz. Note the tendency for epochs of near-coincident firing to persist for the duration of the stimulation trains (1000 ms), and the apparent ‘preference’ of this cell pair for input frequencies <16 Hz.

The stimulus-locking properties of metronome cells suggest that spike-timing can be altered for prolonged periods during rhythmic somatosensory stimulation (see Figures 4 and 5). This may create ideal conditions for stimulus-induced synchronisation of multiple metronome cells across the population. Using the same format as Figure 6D, the correlation delay matrices shown in Figure 6E for the same cell pair show that stimulus-locking gives rise to repeated epochs of near-coincident firing closely tied to the stimulation frequency. Moreover, this behaviour persists for the duration of each stimulation train (1000 ms), although with the cessation of stimulus-locking at the termination of the stimulus train, the cell pair rapidly de-correlated and resumed their idiosyncratic firing (cf. Figure 6C). As stimulus locking degrades with increasing stimulation frequencies, especially >20 Hz (correlation delay matrices not shown) so too does the likelihood of synchronisation, thus near-coincident firing appears most prominent for this cell pair for stimulation frequencies <16 Hz (cf. idiosyncratic frequencies ∼12 Hz and ∼14 Hz).

Considered across the population, correlation delay matrices for grouped data are plotted in Figure 7 showing that the population of metronome cells, each with idiosyncratic frequencies, are capable of temporally encoding a variety of stimulation frequencies into sustained ‘packetised’ near-coincident firing. The stimulus-locking preferences for input frequencies <20 Hz considered alongside the decrement in synchronisation likelihood suggests that the population of metronome cells may behave as a series of band-pass filters (≤20 Hz; cf. *individual* cells behaving as band-pass filters – Figure 4) able to broadcast temporally aligned near-coincident activity to the cerebellum, indexed by the underlying frequency of sensory events.

**Figure 7:** Near-coincident firing in metronomes cells is paced by rhythmic sensory stimulation. Following the same format as Figure 6E, correlation delay matrices are shown for grouped data derived from 11 metronome cell pairs tested with the range of stimulation frequencies. Note the tendency for epochs of near-coincident firing closely indexed by the stimulation frequency and the decline of near-coincident firing for input frequencies ≥20 Hz.

### Synaptic integration of metronome cell spike-timing in granule cells

Our analysis suggests that common inhibitory drive can temporally-align metronome cell spike-timing, leading to a synchronised population broadcast of mossy fibre activity to the cerebellum. Prior modelling work has highlighted precise timing of mossy fibre inputs across granule cell dendrites as a requirement to reach spike-threshold [25], [26]. We examined how metronome mossy fibre signals might summate in a simulated granule cell (see Methods), employing real spike-times recorded from a range of metronome cells (n = 10 cells, covering the range of firing frequencies, only ipsilateral hindlimb responsive cells were arbitrarily selected for consistency and to normalise for peripheral conduction delays). In the first of two scenarios, we assumed that the simulated granule cell received convergent mossy fibre inputs with *similar* frequencies on each of 4 dendrites, in contrast to the alternative scenario where convergent input frequencies were dissimilar, instead covering a broad range (note that spiking and inhibition were not included in the simulation). As expected for the similar input scenario, a single stimulus reveals a resonant EPSP pattern, reflecting the auto-correlation of similar frequencies, particularly close to the idiosyncratic frequency of the mossy fibres (∼16 Hz; Figure 8A). In keeping with the stimulus-locking of individual metronome cells, no patterned EPSP summation occurred for stimulation frequencies of 20 Hz and above (only 20 Hz case shown; cf. 24 Hz and above in Figure 4 and inputs >20 Hz in Figures 6 and 7). In our alternative scenario using dissimilar frequencies, a diverse mixture of metronome cells with firing frequencies ranging from 8 to 16 Hz converging onto a single granule cell produced more complex results. In this situation, single stimuli failed to evoke EPSP summation (Figure 8B). Although our JPSTH analysis suggests that single stimuli evoke mass synchronisation across the population (onset latency ∼50 ms; see Figure 6D), it is not guaranteed that all granule cells receiving convergent metronome mossy fibre inputs would experience this, as precise synchronisation depends on the idiosyncratic firing frequencies of the particular mossy fibres reaching each granule cell. During rhythmic stimulation, modest EPSP patterning is evident at 6 Hz and 12 Hz, with highly coincident patterned EPSP summation visible during 18 Hz stimulation, with a similar failure of summation at the highest frequency. The pronounced resonance at 18 Hz is sharply in contrast to the relative lack of resonance at frequencies bordering this (16 Hz and 20 Hz). Although these models are speculative, they suggest that frequency-specific EPSP patterning may occur in individual granule cells and that these properties may emerge as a function particular pattern of idiosyncratic frequency convergence of metronomic mossy fibres.

**Figure 8:** Simulation of EPSP summation arising from near-coincident firing of metronome cells converging in granule cells. The cartoons in **A** & **B** illustrate the input characteristics used for each simulation of averaged EPSP summation in a simulated granule cell, i.e. *similar* or *dissimilar* convergence of metronome mossy fibres. Spike times from a real metronome cell with 16 Hz idiosyncratic firing frequency were fed to each dendrite in **A**, giving rise to resonant patterning of EPSPs at a variety of rhythmic stimulation frequencies (stimulus pulse times indicated by triangles). In **B**, spike times from 4 individual metronome cells, each with differing idiosyncratic firing frequency, were fed into the model. In contrast to **A**, single stimuli did not bring about EPSP summatioan although rhythmic stimulation, particularly at 18 Hz gave rise to resonant EPSP patterning.

## Discussion

Our experiments reveal an unusual spike-time coding strategy driven by inhibition imposed upon highly regular firing in metronomic neurones which in turn form a major mossy fibre input to the cerebellum.

Phase resetting of spike-time by sensory evoked inhibition can produce either spike-time advancements and delays indexed by the arrival time of the inhibition relative to preceding spontaneous spike. This type of biphasic phase response is known as a type II PRC [57] in contrast to type I PRCs where only spike-time delays are seen. Many PRC studies *in vitro* rely on depolarising current or sinusoidal current injection to evoke firing [54], [58], [59]. Our study has the advantage of exploiting rhythmic spontaneous firing and uses an intact sensory pathway to drive inhibition-mediated phase resetting. Although we do not address the mechanisms behind this inhibition, comparison with GABAergic resetting of intrinsic oscillations and spike-timing mechanisms has been reported in subthalamic neurones [18], also in Type A cells of the globus pallidus (Fig. 4 of [19]) and hippocampal pyramidal cells [17] and indeed GABAergic inhibition has a prominent role in the generation and maintenance of oscillatory activity [7], [60], [61]. Our spike-time advancements (extending over two ISIs; approximately 200 ms) are consistent with GABAergic activation of hyperpolarisation-activated cation currents, such as Ih [54]. Computationally, a pool of oscillators at differing frequencies can efficiently represent the passage of time [62] and although inhibitions appear brief-lived (40–50 ms), the ionic mechanisms underlying regular metronome cell firing create a de facto spike-time ‘memory’ of inhibition arrival times, extending over many hundreds of milliseconds (Figures 3 and S1 of [63]). Neurones considered under integrate-and-fire models (which fire solely on the basis of synaptic events) do not show this property, it being instead a property of resonate-and-fire models. Such models rely on sub-threshold oscillations imparting a membrane resonance to the neurone – inputs timed according to the eigenfrequency, or its factors, may bring the cell to spiking threshold. Inhibitory inputs can also produce post-inhibition spiking, via anodal break excitation (Figures 4 and 8 of [64]) suggesting a close correlate between metronome cells and the resonate-and-fire model. Resonance is generally considered in terms of sub-threshold oscillations, although our metronome cells were spontaneously active raising the possibility that spikes and associated after-potentials might serve as an oscillatory ‘internal’ reset mechanism as well as an output signal [see 63]. As highlighted in Figure 2, metronome cells appear to behave as independent neuronal oscillators since their spikes are intimately associated with locally generated periodic voltage oscillations intimately linked to the cell's idiosyncratic frequency. Since we used spikes and LFP from the same electrode it is possible that slow components of the spikes (afterpotentials) contribute to these LFP oscillations as suggested by Buszaki [45]. However, sub-threshold soma-dendritic membrane voltage oscillations also make a direct contribution to local LFP [44] and we interpret the peri-spike voltage oscillations as reflecting these processes. An additional concern surrounds our use of anaesthetic which may have induced regular firing in metronome cells. However, other cerebellar cell types fire with much greater irregularity under the same conditions (see Figure 1F). Our data suggest that metronome cells possess intrinsic pacemaker-like properties which may be underpinned by persistent sodium currents and calcium activated potassium currents leading to membrane resonance [for review see 10] and auto-rhythmic firing [65], [66]. A further limitation of our experiments concerns the use of electrical micro-stimulation of sensory afferents capable of producing highly synchronous afferent volleys. In contrast, natural sensory stimuli may well evoke lower levels of metronome cell population synchrony although rhythmic behaviours such as whisking, sniffing, etc. are likely to produce synchronous afferent input (discussed later). It is also noteworthy that cerebellar Golgi cells recorded in the same preparation show qualitatively similar responses to electrical or air-puff stimulation of the same sensory areas (Figure 8 of [28]).

Ensemble recordings revealed that single sensory evoked inhibitions can briefly synchronise ensembles of metronome cells (Figure 6C and 6D). Comparable behaviour has been observed in Type A globus pallidus cells sharing inhibitory input [19]. Similarly, olfactory bulb mitral cells can form synchronous ensembles when receiving common inhibitory ‘noise’ [67] suggesting a close correlate between our metronome cell synchrony arising via common inhibitory inputs. Across the population, Type II phase-resetting of spike-times may promote temporal alignment between cells; neurones with Type II PRCs receiving common noisy input synchronise more readily than those with Type I PRC [68]. Thus far, we have only considered the response of metronome cells following a single, randomly delivered, sensory evoked inhibition. The large receptive fields of metronome cells suggest they may gather sensory information from many sources including the face and limbs (Figure S1). Vibrissae movements in rats exhibit a range of frequencies from 2–20 Hz with predominant frequencies around 2 Hz, 5–9 Hz and ∼16 Hz [69] similar to licking [4–7.5 Hz 70], rapid sniffing during odour discrimination [see 71] and stereotyped grooming behaviour [2–7 Hz 72]. Moreover, in cats, cerebellar-projecting LRN cells can receive locomotor and/or rhythmic central respiratory inputs [73]. These sources of rhythmic inputs would be expected to generate periodic/rhythmic barrages of inhibition in metronome cells. Rhythmic stimulation in our experiments created a forced-periodic synchronisation that persisted for the duration of the stimulus (1000 ms), bearing a close correlate with periodic stimulation in the resonate-and-fire model [64]. Metronome spike-timing can reliably represent the sensory stimulation frequency and its factors, with maximal spike-time accuracy occurring for frequencies close to the cell's idiosyncratic frequency. Similar spike-time alignment via phase-resetting of intrinsic oscillations and synchronisation of multiple hippocampal principal cells can be induced by rhythmic stimulation of inhibitory inputs at 5 Hz [17], although in that study other frequencies were not examined. Such behaviour suggests that metronome cells can behave in a manner similar to band-pass filters [c.f. 55], [56] and that as a population they broadcast a ‘packetised’ code of sensory input frequency [74], established through brief-lived epochs of synchronisation, to their downstream targets in the cerebellum. However, the reliability of such a code at the single neurone level may be low since stimulus-spike locking can be <1∶1 (see Figure 4 and 5). None-the-less, these limitations might be compensated for at the population level by synchronised ensembles of cells and through the possible anatomical convergence of metronome cell projections upon their downstream targets.

Functionally, our data complement the view that that one of the major roles for inhibition is to determine precise spike-timing [18], [75]. The most numerous targets for metronome cells are cerebellar granule cells, although Golgi cells may also be targeted. Prior modelling work has highlighted precise timing of inputs across granule cell dendrites as a requirement to reach spike-threshold [25], [26]; we examined these issues using the same granule cell model. Although we did not specifically examine spiking (nor was inhibition included) our simulations suggest that metronomic mossy fibres, if converging on individual granule cells, may impart their resonant properties predisposing granule cells to respond favourably at particular input frequencies and thereby creating preferred times for spike generation. In this regard, the spiking output of granule cells is expected to linearly reflect their membrane potential level [25], [76], although the exact timing of granule cell spikes is subject to stochasticity [77]. Alternatively, synchronised metronomic mossy fibre input may be equally well suited to induce NMDA-receptor mediated plasticity [c.f. theta burst stimulation used by 78]. However, metronome cells are not the only source of mossy fibres and we cannot address the question of whether *all* LRN cells are metronomic; in contrast, other mossy fibre types tend to fire at much higher frequencies (>100 Hz) during signalling [25], [35], [37], [79], [80]. Indeed, a subset of metronome cells do show brief-lived high frequency excitations (see Figure S1C, S1D, S1F and S1H). In agreement with our own observations, other studies have described metronome-like mossy fibre terminals in the anterior lobe of decerebrate cats [81]. These mossy fibres discharged regularly at ∼20 Hz and showed spike-time resetting responses initiated by sensory evoked silent periods, identical to our own responses. Taken together, these observations suggest that metronome cells are at least common to both rats and cats and that they may represent a generalised coding scheme of cerebellar mossy fibres.

If metronome cells converge on individual granule cells our data suggest that the tight synchronisation of their activity across multiple dendrites could generate an EPSP profile similar to the higher frequency firing mossy fibre types. Prior investigations have not described granule cell EPSP patterns predicted by our simulations [25], [26], [80], [82] although it is noteworthy that none of these studies employed rhythmic stimulation – our simulations suggest that this is a key requirement to reveal frequency-patterned EPSP summation, in particular, no EPSP patterning is seen when convergent mossy fibre inputs of dissimilar frequency respond to a single stimulus (Figure 8B) so the possibility remains that frequency-patterned EPSP summation is yet to be observed experimentally. Nonetheless, granule cells *in vitro* show membrane resonance around 4–10 Hz and Golgi cells show pacemaker oscillations at similar frequencies [11], [12], [66], whilst Golgi cells *in vivo* may participate in 5–30 Hz oscillatory activity via gap-junction coupling to other Golgi cells [13]. LFP oscillations (7–25 Hz) in the granular layer have been reported in awake monkeys, rabbits and rats during periods of quiet attentiveness or learning [13], [83]–[85] although the origin of these signals remains unclear their frequency range is a very close correlate with metronome cell firing frequencies (∼7–22 Hz). The resonant properties of Golgi cells and granule cells predisposes them to ‘tune-in’ to oscillatory inputs, thus metronome cells may be one of the principal orchestrators of oscillatory sensorimotor information processing at the input stage of the cerebellum.

## Supporting Information

Figure S1 **Characterisation of somatosensory responses in metronome cells.** The PSTHs in **A** and **B** show typical spike-time resetting responses beginning with silent periods only, for an example brainstem unit and cerebellar unit, respectively. Action potential waveforms are inset – note the dual component action potential of the cerebellar units. Similar data are presented in **C** and **D** illustrating responses beginning with short-lasting excitations (SLE; highest bins in each PSTH) for example brainstem and cerebellar units, respectively. The vibrisssal-evoked SLE response shown in **D** consisted of two discrete excitations – see expanded time-base (inset). The bar charts summarise the response likelihoods from each of six routinely tested skin areas (**E** and **F**) **alongside data for onset latencies and durations of resetting responses overall** (**G**) and SLE excitations only (**H**). Note that two bars are presented for vibrissal responses (cf. **D**). PSTH bin-size 10 ms. Error bars represent mean ±2 S.E.M.
(TIF)

Text S1 Widespread, bilateral receptive fields of metronome cells.
(DOC)
